This article has been retracted.

# Novel NAD‐independent *Avibacterium paragallinarum*: Isolation, characterization and molecular identification in Iran

**DOI:** 10.1002/vms3.754

**Published:** 2022-02-19

**Authors:** Sheida Beiranvand, Tohid Piri‐Gharaghie, Behnaz Dehganzad, Faranak Khedmati, Fatemeh Jalali, Mahya AsadAlizadeh, Hassan Momtaz

**Affiliations:** ^1^ Biotechnology Research Center Shahrekord Branch Islamic Azad University Shahrekord Iran; ^2^ Department of Biotechnology Raberashidi University of Tabriz Tabriz Iran; ^3^ Department of Microbiology Faculty of Basic Sciences Rudehen Branch Islamic Azad University Tehran Iran; ^4^ Department of Medical Nanotechnology Faculty of Basic Sciences Golestan University of Medical Science Golestan Iran; ^5^ Department of Biology Faculty of Basic Sciences University of Tehran Tehran Iran; ^6^ Department of Microbiology Shahrekord Branch Islamic Azad University Shahrekord Iran

**Keywords:** Avibacterium paragallinarum, infectious coryza, nicotinamide adenine dinucleotide‐independent, PCR

## Abstract

**Background:**

Infectious coryza (IC) is an invasive upper respiratory disease caused by *Avibacterium paragallinarum* that affects birds, particularly chickens. The objective of this study is to isolate, characterize and molecularly identify the bacterium *A. paragallinarum* in poultry birds, as well as to determine its antibiotic sensitivity and resistance.

**Methods:**

A total of 10 chickens from four different Iranian farms with typical IC symptoms were used in this study. The nasal swabs were streaked onto chocolate agar plates and blood agar plates and incubated at 37°C in 5% CO_2_ for 24 to 48 h. As part of the identification of bacteria, bacteriological observations and polymerase chain reaction (PCR) testing are conducted. The antibiotic sensitivity tests were also performed using the disk diffusion method against *A. paragallinarum* and the prevalence in different farms was determined.

**Results:**

By using biochemical assays and PCR analyses, seven strains of *A. paragallinarum* were isolated from samples of four chicken farms with typical IC clinical signs. Most isolates (4/7) showed the typical requirement for nicotinamide adenine dinucleotide (NAD) and an enriched CO_2_ atmosphere for growth. Three of the seven strains of *A. paragallinarum* were found to be novel NAD‐independent under anaerobic conditions. There was one biochemical biovar identified in terms of carbohydrate fermentation patterns, although changes in maltose carbohydrate fermentation patterns were detected in the No. 5 strain. All isolates were sensitive to gentamicin and spectinomycin. Three novel NAD‐independent strains (Nos.1, 5 and 7) were found to be multidrug‐resistant (MDR) and resistant to at least three classes of antibiotics. There was greater antibiotic resistance in the three NAD‐independent isolates than in normal NAD‐dependent bacteria.

**Conclusion:**

By discovering NAD‐independent forms of *A. paragallinarum*, these species have a greater range than previously believed. A clear, cautious approach should be taken in diagnosing and possibly controlling IC.

## Graphical abstract

In this study, we showed that NAD, as a growth factor, increases antibiotic resistance in *Avibacterium paragallinarum* strains isolated from poultry meat.

## 1 INTRODUCTION

Infectious coryza (IC), a disease of the upper respiratory system in chickens, is caused by *Avibacterium paragallinarum* (previously *Haemophilus paragallinarum*) (Ali et al., 2013). The incidence of IC is increasing in many parts of the world, affecting chickens of all ages, both indigenous (native chickens) and laying hens in poultry farms (Paudel et al., 2017). In addition, this disease affects developing hens and layers and is economically significant since it increases culling rates and decreases egg output (by between 10 and ‐40%). (Ali et al., 2013; Crispo et al., 2018; Paudel et al., 2017). In the acute phase of the disease, facial swelling, inflammation of the sinuses and conjunctiva and purulent discharge from the nose characterize the disease (Crispo et al., 2018). Beach et al. thought of IC as a separate clinical entity as early as 1920. The common etiological agent was unknown for many years because the disease was frequently misdiagnosed in mixed infections, particularly with chicken pox (Blackall et al., 1997). *Bacillus hemoglobinophilus coryzae gallinarum* was named after the causal agent by DeBlieck (1932) (Blackall et al., 1997). The binomial *Haemophilus gallinarum* was proposed by both Elliot and Lewis and Delaplane et al. in 1934 (Schalm & Beach, 1936). Due to its demand for both x‐(haemin) and v‐(nicotinamide adenine dinucleotide, NAD) factors for development, the causal agent of IC was identified as *H. gallinarum* during research done in the 1930s (Feberwee et al., 2019).

IC is a major economic challenge in many regions of the world. The infection is most prevalent in California and the South‐eastern states of the United States (Blackall et al., 1997). IC is probably available all around the world. Acute catarrhal inflammation of the nasal passages and sinuses is caused by *A. paragallinarum*. Catarrhal conjunctivitis and subcutaneous oedema of the face and wattles are common occurrences. Pneumonia and airsacculitis are uncommon in broilers; nevertheless, certain reports of prevalence in broilers have revealed high levels of contamination (up to 69.8%) due to airsacculitis, even without other viral or bacterial infections (Muhammad & Sreedevi, 2015). At present, there is no definitive treatment available for this condition, and antibiotics can only reduce the severity of the symptoms, and they cannot remove bacteria, so once the antibiotic is stopped, the disease will recur (Jeong et al., 2017).

The use of vaccinations helps to prevent and control infectious diseases such as coryza. In spite of immunization, there is still a risk of acquiring the disease (Deshmukh et al., 2015). It is possible to identify and isolate the causal agent based on symptoms, post‐mortem findings and bacteriological tests of the causative agent, thereby enabling diagnosis (Vargas & Terzolo, 2004). Most isolates of *A. paragallinarum* require NAD as a growth factor (Badouei et al., 2014). NAD‐independent isolates and isolates with unusual growth properties have been identified as well. The inability to ferment d‐xylose and trehalose, as well as the lack of catalase, differentiates *A. paragallinarum* from the other *Avibacterium* species (Badouei et al., 2014). The diagnosis is made based on clinical symptoms, and the confirmation is made by biochemical testing. A rapid, accurate and precise diagnosis using polymerase chain reaction (PCR) is fundamental for avoiding coryza damage (Nouri et al., 2020). The prevalence of the disease has increased from 14 to 25% in recent years, prompting global preventative efforts (Han et al., 2016). Coryza instances increased significantly in California in 2017, according to the California Animal Health and Food Safety Laboratory System, and adequate herd vaccination and biosafety standards should always be established and updated based on these findings. However, there is no specific information on the prevalence of this disease in Iran (Banani et al., 2007). The Razi Institute (Nouri et al., 2020) provided the latest information on the disease diagnosis in 2020. Meanwhile, clinical symptoms of suspected IC are common in Iranian commercial poultry, and treatment with various medicines is done without completing an antibiogram and imported IC vaccination is widely used. However, research on IC and its agent is rare in Iran, with just a few reports of IC agent isolation and identification (Ahmadi & Nasri, 2018; Banani et al., 2007; Nouri et al., 2020). The present study aimed to isolate, molecularly identify and investigate the biochemical properties and antibiotic susceptibility of *A. paragallinarum* bacteria.

## 2 MATERIALS AND METHODS

### 2.1 Ethical consideration and origin of the sample collection

All animal protocols were performed in accordance with the Ethical Committee and Research Deputy of the Islamic Azad University of Shahrekord Branch, Iran for the Care and Use of Laboratory Animals and were approved by the Institutional Animal Care and Use Committee guidelines of Islamic Azad University, Shahrekord, Iran (14th 2020 with ethics code: IR.IAU.SHK.REC.1400.035). The isolates were from probable IC outbreaks on four Iranian commercial broiler breeder and layer farms in various parts of Shahrekord and Isfahan (Iran). The illness was seen in flocks of various ages (18–89 weeks) and breeds. There were symptoms of severe respiratory distress including nasal discharge and a significant decrease in egg production. Egg production losses ranged from 2 to 74%. Twenty submissions of 10 birds from these four farms with clinical symptoms indicative of IC were sent to Lactofeed Company Diagnostic Laboratory (Shahrekord, Iran) for post‐mortem examination and laboratory diagnoses. A total of 20 choanal swabs from backyard chicken cases suspected of IC infection were acquired and transferred to BHI broth media enriched with 0.0025 mg/mL NAD. The collected samples were cultured in the laboratory for less than 2 h to avoid any bacterial inactivation.

### 2.2 Bacterial isolation and culture

A total of 20 choanal swabs from backyard chicken cases suspected of IC infection were acquired and transferred to BHI broth media enriched with 0.0025 mg/mL NAD. The collected samples were cultured in the laboratory for less than 2 h to avoid any bacterial inactivation. Samples were grown on chocolate agar plates for 24 to 48 h at 37°C under 5% CO_2_ with a nurse culture of *Staphylococcus epidermidis* ATCC 14990, whether NAD‐dependent or not. NAD‐dependent *A. paragallinarum* appeared adjacent or next to the nurse culture (satellite phenomenon). Both NAD‐dependent (from chocolate agar) and NAD‐independent colonies (non‐satellite growth on chocolate agar, when present), with the typical *A. paragallinarum* morphology as specified above, were tested for biochemical identification (Xu et al., 2019).

### 2.3 Identification of *A. paragallinarum*

#### 2.3.1 Biochemical identification

For initial identification, the colony with satellite development was stained with Gram staining and evaluated for catalase, oxidase, urease and carbohydrate fermentation using the Gram staining technique. *Avibacterium paragallinarum* is distinguished from other *Avibacterium* species by its inability to ferment both d‐xylose and trehalose and the absence of catalase (Fauziah et al., 2021).

#### 2.3.2 Molecular identification

(A) Primer design: A PCR assay was used to identify and validate the isolated bacteria using 16SrRNA specific primers developed for the genus *A. paragallinarum*. The approved sequence of *A. paragallinarum* species 16S ribosomal RNA gene (AY498868.1) was obtained and utilized for this purpose using the GenBank database (National Center for Biotechnology Information; http://www.ncbi.nlm.nih.gov). The primers of this research were designed with Primer Express bioinformatics software (www.fishersci.se) (Table 1). The validation of the selected primers was performed using BLASTn online tools (GenBank, NCBI, USA) and the Sequence Match program from the Ribosomal Database Project (RDP II, USA). Then the primer designed by Sinaclon (Iran) was synthesized.
(B) DNA extraction and PCR reaction: Briefly, DNA was extracted from isolates by lysing bacterial cells by boiling method. Briefly, the bacterial pellets were suspended in 200 μL of TE buffer (Tris‐HCl [10 mM]: EDTA [1 mM]) for 15 min and then boiled. The sterile Eppendorf tubes were immediately immersed in an ice bath for 15 min after boiling and then centrifuged at room temperature for 5 min at 14,000 rpm. The DNA‐containing supernatant (100 μL) was transferred to a separate sterile tube and kept at –20°C (Junior et al., 2016). PCR amplification was then performed using the Yekta Tajhiz Azma PCR Kit (YTA, Iran) under the following conditions: denaturation at 95°C for 5 min, followed by 30 cycles at 95°C for 1 min, 60°C for 1 min, 72°C for 1 min and a final extension at 72°C for 5 min. *Avibacterium paragallinarum* ATCC 29545 was used as a positive control. DNA‐free microtubes were used as negative controls. A nanodrop device (NanoDrop ND‐2000 Spectrophotometer, NanoDrop Technologies, Wilmington, DE, USA) was used to quantify the quality as well as to quantify the extracted DNA. In this method, the qualitative properties of DNA are determined by reading the ratio A260/A280, in which the amount of light absorption for DNA at a wavelength of 260 nm is measured and the amount of DNA is determined. The best‐case scenario for OD260/OD280 is around 1.8‐2, with values less than 1.8 indicating protein contamination and other UV absorbers. A ratio of more than 2 indicates high RNA in the sample.

**TABLE 1:** The primers of this research were designed with Primer Express software

Reference gene	Sequence (5′ → 3′)	Tm (°C)	Product length (bp)	Volume
*16S ribosomal RNA*	F: ATTCCACGTGTAGCGGTGAA	60	165	25 μL
	R: AGCCCAATCCCCAAATCGAC			

### 2.4 Antimicrobial susceptibility testing

The antimicrobial sensitivity test was carried out utilizing the Chukiatsiri et al. (2012) technique, with minor modifications. *Avibacterium paragallinarum* isolates were screened against the most widely used antibiotic disc. The bacteria suspension was adjusted to a turbidity of 0.5 McFarland standard before being distributed onto Mueller–Hilton Agar medium using a sterile swab. The antimicrobials tested were as follows: gentamicin (10 μg), spectinomycin (100 μg), imipenem (10 μg), tetracycline (10 μg), piperacillin‐tazobactam (100 +10 μg) and ceftazidime (30 μg). The medium was incubated in a 5% CO_2_ incubator at 37°C. Observation of the inhibition zone was made after 24 h and the diameter of the inhibition zone was determined and recorded in millimetres. The susceptibility classification (sensitive, intermediate or resistant) was evaluated by CLSI M61.

### 2.5 Statistical analysis

According to the chi‐square test and Fisher's exact test, there were significant differences among serological surveys based on the year the survey was conducted and the age of the animals. A one‐way ANOVA was performed to compare the means of each group, and the Bonferroni correction was applied for multiple comparisons, to compare the clinical sign ratings of the experimental groups. For all analyses, a *p* < 0.05 was deemed statistically significant.

## 3 RESULTS

### 3.1 Case history

As shown in Table 2, efforts to isolate *A. paragallinarum* were performed by swabbing the infraorbital sinus of birds from poultry farms with a history of reduced egg production.

**TABLE 2:** Detailed description of post‐mortem examination (PME) of *A. paragallinarum* isolates involved in clinical outbreaks of infectious coryza

Farm	Breed	Number of chickens	Gross lesions	Origin
A	Broiler breeder	10	Enlargement of bottom of jaw, parasites in intestine, Nasal discharge.	Shahrekord
B	Broiler breeder	10	Airsacculitis, haemorrhage in larynx, Nasal discharge.	Isfahan
C	Layer	10	Mucous increase in upper respiratory organ, Oedema or swelling of the face	Shahrekord
D	Layer	10	Mucous increase in upper respiratory organ, Oedema or swelling of the face	Isfahan

Swelling of the infraorbital sinus, oedema of the surrounding tissues, occasionally spreading to the wattles and hyperaemia of the conjunctiva are all common findings in the instances that were presented. Eyelid and wattle oedema ranged from severe to minor (Figure 1).

**FIGURE 1:** The proportion of signs of chickens infected with different *A. paragallinarum* isolates. (a) Oedema or swelling of the face. (b) Nasal discharge observed

### 3.2 Bacterial isolation and biochemical identification

Information about the appearance of bacteria and bacterial colonies on solid culture media (chocolate agar plates) is given in this field (Figure 2). The appearance of clear, dew‐like colonies on chocolate agar indicated the field strain of *A. paragallinarum*. Co‐culture of strains suspected of *A. paragallinarum* with *S. epidermidis* ATCC 14990 also showed larger colonies close to the *Staphylococcus* line. This indicates haemolysis and release of factor V from red blood cells by *Staphylococcus*, which results in increased growth of *A. paragallinarum* and is an initial confirmation of *A. paragallinarum* isolation.

**FIGURE 2:** *Avibacterium paragallinarum*, cultivated for 48 h at 37°C in 5% CO_2_ on haematin agar (choclate agar). Because this bacterium does not grow well on regular blood agar, it is usually grown on haematin agar, where the colonies may be seen. (a) *Avibacterium paragallinarum* grow on choclate agar. (b) Clear dew‐like colonies of *A. paragallinarum* in chocolate agar. (c) *A. paragallinarum*, cultivated together with *Staphylococcus epidermidis* ATCC 14990. (d) *A. paragallinarum* has grown in size, forming larger colonies along the *S. epidermidis* ATCC 14990 streak, which causes haemolysis and the release of the V factor from erythrocytes

Seven field isolates were obtained and identified as *A. paragallinarum* using Gram staining, and biochemical testing between 2020 and 2021 (Table 3). All of the isolates were Gram‐negative, catalase‐deficient and could not grow on MacConkey agar. d‐mannitol, maltose generated acid in all strains, but not d‐xylose or trehalose (Table 3). Variable acid generation from maltose and d‐xylose was observed, allowing three biochemically unique biovars to be identified based on carbohydrate fermentation patterns. However, differences in maltose carbohydrate fermentation patterns were discovered in the No. 5 strain. The majority of the isolates (4 of 7) needed NAD and 5% CO_2_, but three of them (Nos.1, 5 and 7) were NAD‐independent and developed on blood agar in anaerobic conditions.

**TABLE 3:** Characterization of seven field isolates of *A. paragallinarum*

							Carbohydrate fermentation pattern			
Number	Shape	NAD requirement	Growth in Air	Catalase	Oxidase	Urease	Maltose	d‐ Xylose	d‐mannitol	Trehalose
1	Coccobacillus	−	−	−	−	+	+	−	+	−
2	Coccobacillus	+	+	−	−	−	+	−	+	−
3	Coccobacillus	+	−	−	−	−	+	−	+	−
4	Coccobacillus	+	+	−	−	−	+	−	+	−
5	Coccobacillus	−	−	−	−	+	−	−	+	−
6	Coccobacillus	+	+	−	−	−	+	−	+	−
7	Coccobacillus	−	−	−	−	+	+	−	+	−
ATCC 29545	Coccobacillus	+	−	−	−	−	+	−	+	−

### 3.3 Molecular identification of *A. paragallinarum*

Primers were designed for this study using Primer Express bioinformatics software. The forward and reverse primers of Table 2 were identified as specific primers for *A. paragallinarum*. The designed primers were first evaluated using the BLASTn tool, which identified the high specificity of primer sequences designed for the genus *A. paragallinarum* based on the results of 100 different isolates of *A. paragallinarum* with Query Cover equals to 100% and percent identity score equals 100%. The presence of an expected 165 bp band in electrophoresis of their species‐specific PCR results verified the molecular detection and identification of these isolates (Figure 3). According to the results of PCR and biochemical tests, seven different strains of *A. paragallinarum* were identified and used for antimicrobial sensitivity.

**FIGURE 3:** Molecular identification of *A. paragallinarum* in samples by PCR. M: marker 100 bp‐plus (YTA, Iran); C‐: negative control. C+: positive control, *A. paragallinarum* ATCC 29545 (165 bp); Lane 1, 2, 3, 4, 5, 6 and 7: the positive samples with 165 bp band

### 3.4 Antimicrobial susceptibility

An antibiogram test was used to evaluate antimicrobial susceptibility. According to the antibiotic susceptibility Table 4, all seven *A. paragallinarum* strains were susceptible to gentamicin and spectinomycin (100%). The results of this test showed that one, five and seven bacterial strains are resistant to more than three antibiotic classes, so that these bacteria are a subset of multi‐drug resistant (MDR) bacteria. The pattern of antibiotic resistance of the tested strains is recorded in Table 4.

**TABLE 4:** Summary of antibiotic sensitivity test against seven field isolates of *Avibacterium paragallinarum* using the disk diffusion test

	Aminoglycosides		Carbapenem	Inhibitor	Antibiotics + inhibitors	Cephalosporins	
Strain/symbol	GEN (mm)	SPC (mm)	IMI (mm)	TET (mm)	PTZ (mm)	CAZ (mm)	Phenotype
1	S (16)	S (18)	R (12)	R (14)	R (15)	R (11)	MDR**
2	S (17)	S (17)	I (18)	I (20)	I (19)	S (18)	Non‐MDR
3	S (16)	S (17)	I (19)	S (21)	I (18)	I (16)	Non‐MDR
4	S (18)	S (18)	I (18)	I (19)	I (21)	S (18)	Non‐MDR
5	S (15)	S (17)	R (13)	R (13)	R (12)	R (12)	MDR**
6	S (17)	S (19)	I (21)	S (21)	I (18)	I (17)	Non‐MDR
7	S (17)	S (17)	R (14)	R (14)	R (13)	R (10)	MDR**
ATCC 29545	S (18)	S (17)	S (22)	S (24)	S (23)	S (19)	Non‐MDR
Detection range	S: ≥15	S: ≥17	S: ≥22	S: ≥21	S: ≥21	S: ≥18	S = sensitive
	R: 12 ≥	R: 14 ≥	R: 18≥	R: 17≥	R: 17 ≥	R: 14 ≥	R = resistant
							I = Intermediate

### 3.5 Prevalence assessment

In *A. paragallinarum* species‐specific PCR assays, 35 out of 40 (87.5%) of examined birds were found to be infected with the *A. paragallinarum*. Furthermore, out of 20 broilers (10 farm chickens A and 10 farm chickens B) suspected of coryza, 16 chickens (80%) were positive for *A. paragallinarum*. However, in the Layer chicken group, out of a total of 20 farm chickens C and D, 19 chickens (95%) were positive for *A. paragallinarum*. Farm B with seven (70%) positive sample of *A. paragallinarum* showed less infection than Farm A with 9 (90%). Furthermore, farm C with 10 (100%) positive sample of *A. paragallinarum* showed more infection than farm D with 9 (90%) positive sample (Figure 4).

**FIGURE 4:** *Avibacterium paragallinarum* prevalence in the research groups. (a) *Avibacterium paragallinarum* prevalence in Broiler breeder and Layer groups (b) *Avibacterium paragallinarum* prevalence in Broiler breeder and Layer groups in various farms

## 4 DISCUSSION

IC has a nearly worldwide distribution, and to our knowledge, there is little information on the disease's precise frequency among industrial breeder flocks and/or backyard poultry in Iran (Badouei et al., 2014). The persistence of the IC agent among chicken farms is thought to be due to multi‐age poultry manufacturing systems, partial immunity provided by serovar content in commercial vaccines against regionally prevalent *A. paragallinarum* serovars, and the role of backyard chicken as a source of IC infection for nearby chicken flocks (Gallardo et al., 2020). In spite of occasional reports of IC from Iran, no molecular surveillance data are available to describe the epidemiology of the disease in our surrounding nations (Badouei et al., 2014). Officially, no cases of IC have been documented in Iranian commercial poultry flocks, which might be a favourable result of imported vaccine immunization procedures against serogroups A, B and C throughout the previous decades (Ahmadi & Nasri, 2018; Badouei et al., 2014; Banani et al., 2007; Nouri et al., 2020). However, in recent years, a clinical picture of IC has been described informally in certain layer farms. Vaccinations used in the most sensitive poultry flocks, such as layer and breeder chickens, appear to have brought IC in chicken farms under control (Luna‐Galaz et al., 2016). In the meantime, poultry veterinarians are having difficulty diagnosing poultry illnesses in rural areas and live bird markets (Gharaghie & Shandiz, 2018; Nouri et al., 2020). As a result, we attempted to extract *A. paragallinarum* from hens exhibiting clinical signs of IC, such as oedema in the face and wattle, as well as a reduction in egg production. The birds used in this study were between the ages of 18‐ and 89‐week‐old and came from four farms in central Iran, each with about 10 birds. The isolation of seven *A. paragallinarum* was based on bacterial culture results from 20 swab specimens collected from each likely group of birds. All isolates were V‐factor dependent, showing typical ‘satellite’ growth on solid plate cultures. Consistent with other studies (Ahmadi & Nasri, 2018; Badouei et al., 2014; Banani et al., 2007; Blackall & Soriano‐Vargas, 2020; Blackall et al., 1990; Falconi‐Agapito et al., 2015; Gallardo et al., 2020; Han et al., 2016; Luna‐Galaz et al., 2016; Nouri et al., 2020; Vargas & Terzolo, 2004), the result of the biochemical identification method was the isolation of Gram‐negative, catalase‐negative, oxidase‐negative coccobacilli, which were d‐xylose and trehalose‐negative in fermentation, but were able to ferment d‐mannitol and maltose. These are some of the biochemical features of bacteria that cause IC (Blackall & Soriano‐Vargas, 2020). However, differences in maltose carbohydrate fermentation patterns were discovered in the No. 5 strain. The majority of the isolates (4 of 7) needed NAD and 5% CO_2_, but three of them (Nos.1, 5 and 7) were NAD‐independent and developed on blood agar in anaerobic conditions. This is the only research that we are aware of that reports the identification of various *A. paragallinarum* growth variations in Iran. NAD‐independent *A. paragallinarum* isolates have been found in South Africa, Mexico and Peru thus far (Falconi‐Agapito et al., 2015; Garcia et al., 2004). The two NAD‐independent isolates in this investigation were from two separate commercial layer farms and one from a broiler breeder farm, with three of them coming from probable IC cases that had been treated with antibiotics. *A. paragallinarum* was verified by PCR using 16S ribosomal RNA‐specific primers. PCR assays can be used to simplify the diagnostic process after initial isolation and biochemical identification (Badouei et al., 2014). Another benefit of this procedure is its quickness since the findings are available in less than 24 h. The PCR method was utilized to diagnose coryza in chickens in this study. All seven of the suspicious isolates acquired from culture produced the *A. paragallinarum* unique band (165 bp). The efficacy of accurate identification of IC purely based on culture method from a choanal cleft in naturally infected chicken is reflected in the biochemical method's result when compared to PCR detection. This finding is similar to Chen et al. (1996), who found that PCR testing in natural conditions returned 15 of 39 birds and 6 of 8 commercial farms positive, compared to 8 of 39 birds and 4 of 8 commercial farms positive via culture (Chen et al., 1996). The importance of diligent, continuing monitoring of *A. paragallinarum* isolates is highlighted by the variability in antibiotic sensitivity patterns between isolates from different countries (Luna‐Galaz et al., 2016; Nhung et al., 2017). There is very little information on isolation and antibiotic susceptibility of *A. paragallinarum* prevalence in Iran and is limited to the report of Banani et al. (2007) and Nouri et al. (2020). This analysis confirmed that all *A. paragallinarum* strains were sensitive to gentamicin and spectinomycin, as reported by Nouri et al. Three novel NAD‐independent strains (Nos.1, 5 and 7), are described as the first MDR strains from Iran in this investigation, showing resistance to at least three classes of antibiotics. Various antibiotics showed high and moderate resistance to the bacteria, according to reports from other countries (Chukiatsiri et al., 2012; Priya et al., 2012). Previous research suggests that NAD‐independent isolates may be able to escape host immunological responses, which might result in vaccination failure if the vaccine is based on a NAD‐dependent *A. paragallinarum* strain (Bragg et al., 1997; Jeong et al., 2017). However, the relevance of NAD‐independent isolates in vaccination failures is unclear, as a commercial trivalent vaccine based on typical NAD‐dependent strains has been found to protect against challenge by NAD‐independent isolates under experimental conditions (Jacobs & Van der Werf, 2000). Diagnostic laboratories must also be aware of the possibility of *A. paragallinarum* strains that are not dependent on NAD. *Ornithobacterium rhinotracheale*, another catalase‐negative, Gram‐negative bacterium, might readily be mistaken for these NAD‐independent isolates (Jeong et al., 2017). A serological study of flocks positive for *A. paragallinarum* indicated high positivity rates of 86.4% in 2009, 78.9% in 2010, 70.0% in 2011 and 69.6 % in 2012 (Han et al., 2016; Siddique et al., 2012). In contrast, *A. paragallinarum* was found to be present in 87.5% of samples suspected of being infected with IC in the current investigation, which indicates the high prevalence of *A. paragallinarum*.

## 5 CONCLUSIONS

Using biochemical assays and PCR analyses, seven strains of *A. paragallinarum* were isolated from samples of four chicken farms with typical IC clinical signs. Three of the seven strains of *A. paragallinarum* were found to be NAD‐independent and MDR. In this study, the isolation, identification and antibiotic pattern of *A. paragallinarum* are critical in providing options for coryza disease control. Reports from field cases indicate that commercial vaccines have not been able to cover the prevalence of IC in Iran. While screening for antibiotic susceptibility, provides a beneficial suggestion for an appropriate therapy that is successful and efficient against bacterial infection. Molecular characteristics of *A. paragallinarum* obtained using PCR aid in the rapid diagnosis of these bacteria. The frequency of *A. paragallinarum* in broiler and layer hens in Iran was found to be 87.5% in the current investigation. To rule out the existence of *A. paragallinarum* in chickens in Iran, more study with bigger sample sizes and better sampling methods is needed in different seasons and geographical locations.

## CONSENT FOR PUBLICATION

Not applicable.

## CONFLICT OF INTEREST

The authors declare that they have no conflict of interest.

## ETHICS STATEMENT

The research was extracted from the research project in the field of Microbial biotechnology and was ethically approved by the Council of Research of the Faculty of Basic Science, Shahrekord Branch, Islamic Azad University, Shahrekord, Iran. Verification of this research project and the licenses related to sampling process were approved by the Prof. Hassan Momtaz (Approval Ref Number MIC201946).

## AUTHORS’ CONTRIBUTIONS

**Sheida Beiranvand**: Investigation; Methodology. **Behnaz Dehganzad**: Methodology; Validation. **Faranak Khedmati**: Investigation; Software. Fatemeh Jalali: Funding acquisition; Project administration. **Mahya AsadAlizadeh**: Writing–original draft; Writing–review & editing.

### PEER REVIEW

The peer review history for this article is available at https://publons.com/publon/10.1002/vms3.754

## Data Availability

All data analysed during this study are included in this published article.
